The article "Asymptomatic subjects with diabetes have a comparable risk of coronary artery disease to Non-diabetic subjects presenting chest pain: a 4-year community-based prospective study" was published in 2013. Journal: BMC Cardiovasc Disord.

# Asymptomatic subjects with diabetes have a comparable risk of coronary artery disease to Non-diabetic subjects presenting chest pain: a 4-year community-based prospective study

**DOI:** 10.1186/1471-2261-13-87

**Published:** 2013-10-18

**Authors:** Bo Kyung Koo, Yun Gi Kim, Kyong Soo Park, Min Kyong Moon

**Affiliations:** 1 Department of Internal Medicine, Seoul National University College of Medicine, 39 Boramae Road, Seoul, Dongjak-Gu 156-707, South Korea; 2 Department of Internal Medicine, Boramae Medical Center, Seoul, South Korea

**Keywords:** Diabetes, Coronary artery disease, Chest pain

## Abstract

**Background:**

Although diabetes mellitus is an important risk factor of coronary artery disease (CAD), routine screening for CAD is not recommended for asymptomatic diabetic patients. We assessed the impact of chest pain on CAD risk according to the presence or absence of diabetes mellitus.

**Methods:**

We investigated the future CAD event rate in subjects with and without chest pain according to the presence or absence of diabetes in a prospective large-scale community-based study in Korea.

**Results:**

Among 8,574 subjects (4,032 men and 4,542 women) without a history of CAD, 0.8% and 2.2% of non-diabetic and diabetic subjects, respectively, reported newly developed CAD events during 4 years of follow-up. Although the presence of chest pain at baseline was also significantly associated with an increased risk of CAD of more than 2-fold in both non-diabetic and diabetic subjects (*P* < 0.01), the risk of future CVD event in asymptomatic diabetic patients was not significantly different from that in non-diabetic subjects with chest pain (hazard ratio, 0.907; 95% confidence interval, 0.412 – 1.998).

**Conclusions:**

The CAD event rate of asymptomatic subjects with diabetes was comparable to that of non-diabetic subjects reporting chest pain. Considering the high risk of CAD in asymptomatic diabetic patients, more clinical trials aimed at formulating strategies to screen asymptomatic diabetic subjects should be carried out.

## Background

A large population-based study has suggested that diabetes mellitus is a coronary artery disease (CAD) equivalent [1]. Therefore, it might be very valuable to be able to predict which patients with diabetes will have silent ischemia. However, recent studies have concluded that a conventional risk factor-based approach cannot identify high-risk patients in screening tests [2,3], and that there is no clinical benefit of routine screening of asymptomatic patients with diabetes [2,4]. Furthermore, since recent randomized controlled studies have shown that cardiac reperfusion therapy does not produce better clinical outcomes than medical therapy for stable CAD [5,6], these observations have raised the question of whether or not asymptomatic patients with diabetes should be screened for CAD and experts recommends that candidates for cardiac testing should be limited to those with (i) typical or atypical cardiac symptoms and (ii) an abnormal resting electrocardiogram (ECG) [7].

However, the prevalence of silent myocardial ischemia in asymptomatic diabetic patients with no cardiac history and with a normal 12-lead ECG at rest has been reported to be high (~35%) [8] and such asymptomatic diabetic patients suffer more future cardiac events than symptomatic patients do despite similar coronary atherosclerosis severity [9]. In the Detection of Ischemia in Asymptomatic Diabetics (DIAD) study, a large randomized clinical trial to show no clinical benefit of screening of asymptomatic patients with diabetes, only 15% of subjects classified as having moderate or large perfusion defects underwent coronary angiography within 120 days after screening [4], which might account for the lack of a significant difference between the screened and unscreened groups in that study.

Therefore, we investigated the future CAD event rate in diabetic patients with and without chest pain in a prospective community-based cohort study performed in the Korean population. In addition, we assessed the impact of chest pain on CAD risk according to the presence or absence of diabetes mellitus.

## Methods

### Ansung–Ansan cohort design

The Ansung and Ansan cohorts represent rural and urban areas of Korea, respectively. The design and baseline characteristics of these cohorts have been described elsewhere [10,11]. Briefly, the Ansung–Ansan cohort was established for a prospective large-scale community-based epidemiologic study to investigate chronic diseases in Korea. The eligibility criteria were age 40–69 years old and residence within the borders of the survey areas for at least 6 months before testing. In Ansung, 5,018 of 7,192 eligible individuals were surveyed (70% response rate) using a cluster sampling method stratified by age, sex, and residential district. Ansan is a representative urban community that had a population of 554,998 in 2000 [12]; 5,020 of 15,580 eligible subjects (32.4%) were recruited for the survey through a random sampling method using the local telephone directory. The baseline survey was performed from 2000–2001, and biennial follow-up surveys have been performed since then. Throughout the study, data were collected by the same trained researchers and instruments. Anthropometric parameters and blood pressure were measured by standard methods. The fasting plasma concentrations of glucose, HbA1c, total cholesterol, triglycerides and HDL cholesterol were measured in a central laboratory as described previously [10,11].

Participants completed questionnaires in face-to-face interviews about demographics and previous medical history, including myocardial infarction, heart failure, smoking, medication such as anti-hypertensive drugs or anti-diabetic drugs, and subjective symptoms such as chest pain and dyspnea.

This study was carried out in accordance with the Declaration of Helsinki (http://www.wma.net/en/30publications/10policies/b3/index.html). Informed written consent was obtained from all participants. The study protocol was approved by the ethics committee of the Korean Center for Disease Control and the Ajou University School of Medicine Institutional Review Board.

### Definitions

Cases of diabetes mellitus were defined as subjects who used anti-diabetic medication including insulin at the time of the survey, had HbA1c ≥ 6.5% or 8-hour fasting plasma glucose ≥ 7.0 mmol/L. Hypertension was defined as systolic blood pressure ≥ 140 mmHg, diastolic blood pressure ≥ 90 mmHg, or taking antihypertensive medications. Cases with systolic blood pressure ≥ 140 mmHg or diastolic blood pressure ≥ 90 mmHg were classified as “uncontrolled hypertension.” Dyslipidemia was defined as triglycerides ≥ 1.7 mmol/L after at least 12 hours of fasting, LDL cholesterol ≥ 4.1 mmol/L according to NCEP criteria [13], or taking any lipid-lowering medications. ECG abnormalities suggesting myocardial ischemia at baseline included ST depression ≥ 1.0 mm, T wave inversion ≥ 5.0 mm, ST elevation ≥ 1.0 mm or Q wave at any lead. The definition of a CAD event for next 4 years of follow-up was based on the questionnaire administered in biennial follow-up surveys. Subject with CAD events was defined as subject who answered that they took medication or underwent reperfusion therapy or bypass surgery for any CAD including myocardial infarction. A family history of CAD was defined as when a subject had at least one first-degree relative suffering from CAD. Information about the perception of chest pain according to activity intensity in daily life at baseline was also obtained from the questionnaire. The questionnaire on chest pain comprised questions about the presence of any type of chest pain in daily life, during mild-intensity activity such as walking, and moderate-intensity activity such as climbing stairs. The characteristics of chest pain at each activity level were further categorized as “heaviness,” “tightness or squeezing,” “burning,” “stabbing,” or “lancinating”. Typical angina chest pain of CAD was defined by its characteristics, described as heaviness, tightness, or squeezing.

### Statistical analysis

All data were analyzed by SPSS (SPSS Inc., Chicago, IL, USA). The results are presented as means ± SD. We logarithmically transformed waist circumference, triglyceride concentration, HDL cholesterol concentration, BMI, and urine albumin-to-creatinine ratio for analysis. To determine the significance of differences between baseline clinical characteristics in the development of CAD events during the follow-up period, linear regression and logistic regression analyses adjusted for age were used. In the case of categorical variable, general linear model was used. Cox regression analysis with dummy variables (to contrast the different categories) was used to analyze the hazard ratio (HR) of diabetes and chest pain at baseline for future CAD events adjusted for age, sex and BMI; non-diabetic subjects without chest pain were used as a reference risk group. Hazard function from Cox regression analysis adjusting sex and age were used to construct figures for CAD event according to chest pain and diabetes. The level of significance was set at *P* < 0.05.

## Results

### Baseline characteristics

Of the 10,038 subjects in the Ansung–Ansan cohort, we included 8,574 subjects (4,032 men and 4,542 women) who had no history of ischemic heart disease and no ECG abnormality suggesting myocardial ischemia the present study. Among them, 1,203 (14%) had diabetes mellitus at baseline. During a follow-up period of 4 years, 0.8% and 2.2% of non-diabetic and diabetic subjects, respectively, reported experiencing a newly developed CAD event (Table 1). Among 84 subjects with CAD events during follow-up period, 16 (7 in non-diabetic subjects and 9 in diabetic subjects) reported to have undergone reperfusion therapy in that period. The presence of diabetes at baseline independently increased the risk of future CAD risk (age-, sex-, and BMI-adjusted odds ratio [OR] = 2.083 [95% confidence interval, 1.290 – 3.365], *P* = 0.003). The baseline characteristics according to development of CAD events during the follow-up period are shown in Table 1. Among non-diabetic subjects, those who developed CAD were significantly older (*P* < 0.001), had higher BMI (*P* = 0.001) and waist circumference (WC) (*P* = 0.032 in men and 0.001 in women), and had hypertriglyceridemia more frequently at baseline (*P* = 0.009). However, in diabetic subjects, there were no significant differences between subjects with and without CAD with respect to baseline characteristics, except age (*P* = 0.050). The proportions of all diabetes patients who attained the clinical goals were as follows: 52.0% for HbA1c < 7%, 26.4% for LDL < 2.6 mmol/L, and 76.7% for blood pressure < 140/90 mmHg; none of these parameters differed significantly between those with and without CAD events (Table 1). Age was only a significant risk factor of future CAD events in both men and women in the case of diabetes (data not shown).

**Table 1:** Baseline characteristics of subjects with or without coronary artery disease events over 4 years of follow-up

		**Subjects without diabetes mellitus**			**Subjects with diabetes mellitus**		
		**No CAD at follow-up**	**CAD at follow-up**	***P***^**a**^	**No CAD at follow-up**	**CAD at follow-up**	***P***^**a**^
N (% Men)		7314 (46.5)	57 (40.4)	0.415	1176 (50.9)	27 (48.1)	0.994
Ansung (% Men)		3289 (43.7)	36 (36.1)		595 (43.9)	18 (55.6)	
Ansan (% Men)		4025 (48.7)	21 (47.6)		581 (58.0)	9 (33.3)	
Age (years)		51 ± 9	56 ± 9	<0.001	56 ± 9	59 ± 9	0.050
BMI (kg/m^2^)		24.4 ± 3.1	25.7 ± 2.9	0.001	25.6 ± 3.3	25.5 ± 3.9	0.988
Waist circumference (cm)	Men	83.2 ± 7.5	86.5 ± 6.7	0.032	86.2 ± 8.7	88.5 ± 8.8	0.262
	Women	80.6 ± 9.5	87.4 ± 7.5	0.001	87.1 ± 8.6	86.6 ± 8.8	0.699
Systolic blood pressure (mmHg)		116 ± 18	121 ± 15	0.249	124 ± 19	126 ± 17	0.986
Diastolic blood pressure (mmHg)		74 ± 12	76 ± 9	0.805	77 ± 11	76 ± 10	0.463
HbA1C (%)		5.5 ± 0.3	5.6 ± 0.4	0.758	7.4 ± 1.6	7.1 ± 1.5	0.513
Fasting glucose (mmol/L)		4.7 ± 0.5	4.7 ± 0.4	0.700	6.9 ± 2.6	6.7 ± 2.5	0.986
Total cholesterol (mmol/L)		4.93 ± 0.90	5.21 ± 0.99	0.031	5.21 ± 1.07	5.01 ± 1.10	0.402
HDL cholesterol (mmol/L)	Men	1.16 ± 0.27	1.25 ± 0.38	0.327	1.11 ± 0.26	1.15 ± 0.29	0.630
	Women	1.24 ± 0.28	1.22 ± 0.31	0.865	1.14 ± 0.27	1.17 ± 0.23	0.600
Triglyceride (mmol/L)		1.68 ± 1.06	1.95 ± 0.99	0.032	2.31 ± 1.52	2.07 ± 0.96	0.634
Serum creatinine (μmol/L)		74 ± 18	72 ± 14	0.506	76 ± 37	80 ± 28	0.551
Urine microalbuminuria(mg/g Cr)		97 ± 244	79 ± 60	0.665	180 ± 487	182 ± 191	0.623
Normal (%)		17.2	8.7		10.6	0.0	
Microalbuminuria (%)		79.3	91.3	0.424	79.4	80.0	0.475
Proteinuria (%)		3.0	0.0		10.0	20.0	
Smoker							
Non-smoker (%)		59.9	57.9		56.2	53.3	
Ex-smoker (%)		15.1	17.5	0.591	16.8	16.7	0.631
Smoker (%)		25.0	24.6		27.0	30.0	
Family history of CAD, N (%)		22 (0.3%)	0 (0)	0.998	2 (0.2)	0 (0)	1.000
Hypertension, N (%)		1355 (18.5)	19 (33.3)	0.074	425 (36.1)	14 (51.9)	0.237
Antihypertensive drug, N (%)		591 (8.1)	14 (24.6)	0.001^c^	260 (22.1)	11 (40.7)	0.090
Hypertension, uncontrolled, N (%)^b^		990 (13.5)	9 (15.8)	0.393	274 (23.3)	6 (22.2)	0.237
Dyslipidemia, N (%)		3051 (41.7)	34 (59.6)	0.016^d^	786 (66.7)	18 (66.7)	0.959
Cholesterol-lowering drug, N (%)		20 (0.3)	0	0.998	15 (1.3)	0	0.998
Triglyceride ≥ 1.7 mmol/L, N (%)		2627 (35.9)	31 (54.4)	0.009^e^	721 (61.5)	17 (63.0)	0.813
LDL cholesterol < 4.1 mmol/L, N (%)		6562 (89.7)	52 (91.2)	0.672	959 (81.8)	22 (81.5)	0.887
LDL cholesterol < 3.3 mmol/L, N (%)		4860 (66.5)	38 (66.7)	0.870	672 (57.3)	18 (66.7)	0.379
LDL cholesterol < 2.6 mmol/L, N (%)		2212 (30.2)	17 (29.8)	0.967	306 (26.1)	11 (40.7)	0.116
HbA1c < 7%, N (%)		-	-	-	609 (51.8)	16 (59.3)	0.423
Living in urban area (Ansan) (%)		51.4%	33.3%	0.150	46.5%	30.0%	0.622

*Abbreviations*: CAD, coronary artery disease.

^a^Age-adjusted *P* value; ^b^Cases with systolic blood pressure ≥ 140 mmHg or diastolic blood pressure ≥ 90 mmHg irrespective of medication; ^c^Odds ratio (OR) for CAD = 2.829 [1.501- 5.333]; ^d^OR = 1.928 [1.132 – 3.285]; ^e^OR = 2.014 [1.192 – 3.404].

### CAD event rate according to the presence or absence of chest pain

At baseline, 22.8% and 19.6% of non-diabetic and diabetic subjects, respectively, reported having any type of chest pain in daily life. Approximately 40% of subjects with CAD events previously reported chest pain at baseline irrespective of glycemic status. Among all subjects reporting chest pain at baseline, 1.6% and 5.1% of non-diabetic and diabetic subjects, respectively, experienced CAD events over the next 4 years. The presence of chest pain at baseline was significantly associated with a 2-fold increase in future CAD risk in both non-diabetic (HR = 2.879 [1.536 – 5.394], *P* = 0.001) and diabetic subjects (OR = 3.489 [1.620 – 7.512], *P* = 0.001) even after adjusting for sex and age (Table 2). Exertional chest pain during mild-degree exercise was also a significant predictive factor of CAD events in non-diabetic subjects (Table 2). In contrast, there was no significant association between chest pain during mild-degree exercise and the CAD event rate in diabetic subjects.

**Table 2:** Hazard ratios (HR) of CAD events during next 4 years according to the perception of chest pain at baseline

		**Subjects without diabetes mellitus**				**Subjects with diabetes mellitus**			
		**Number of cases**	**CAD at follow-up (1000 person-yr)**	**Hazard ratios**^**a**^	***P***^**b**^	**Number of cases**	**CAD at follow-up (1000 person-yr)**	**Hazard ratios**^**a**^	***P***^**b**^
Chest pain, total (%)									
	Absence	5624	1.0	2.879	0.001	959	3.9	3.489	0.001
	Presence	1674	2.7	(1.536 – 5.394)		235	13.0	(1.620 – 7.512)	
Typical chest pain (%)^c^									
	Absence	6596	1.1	2.814	0.005	1084	4.6	3.279	0.007
	Presence	779	3.2	(1.370 – 5.780)		120	15.0	(1.380 – 7.793)	
Chest pain on mild-intensity activity (%)^d^									
	Absence	7146	1.2	6.110	0.003	1171	5.6	1.904	0.530
	Presence	94	8.2	(1.861 –20.054)		19	13.3	(0.255 – 14.222)	
Chest pain on moderate-intensity exercise (%)^d^									
	Absence	7067	1.3	2.017	0.338	1158	5.2	3.926	0.028
	Presence	192	2.7	(0.480 – 8.472)		33	23.8	(1.162 – 13.265)	

*Abbreviations*: CAD, coronary artery disease.

^a^Hazard ratio of chest pain for CAD events over the next 4 years adjusting sex and age; ^b^sex- and age- adjusted *P* value; ^c^chest pain described as heaviness, tightness, or squeezing regardless of activity level or chest pain perception; ^d^any chest pain associated with activity.

Next, we estimated HR of CAD events according to presence or absence of chest pain in the subjects with or without diabetes using Cox proportional hazards model. All study subjects were categorized into 4 groups: non-diabetic subjects without chest pain at baseline (Group 1), non-diabetic subjects with chest pain (Group 2), diabetic subjects without chest pain (Group 3), and diabetic subjects with chest pain (Group 4). Group 4 had the worst prognosis, whereas Group 1 had the best (Figure 1). Groups 2 and 3 had intermediate event rates as well as similar outcomes. Table 3 presents the results of the Cox proportional hazards model comparing the subjects in Groups 2–4 with those in Group 1. Groups 2–4 had significantly higher HRs than Group 1 even after adjusting for age, sex, and other risk factor of CAD. Next, we compared only Groups 2 and 3. The age- and sex-adjusted HR of Group 3 was not significantly different from that of Group 2 (HR = 0.907 [0.412 – 1.998], *P* = 0.809), suggesting these groups have similar CAD event rates.

**Figure 1:** **Cox proportional hazards model for the probability of coronary artery disease (CAD) events over the 4 years.** Cox proportional hazards model for the probability of CAD events in 1,203 subjects with diabetes mellitus and 7,371 non-diabetic subjects with and without chest pain at baseline. Gray dotted line, non-diabetic subjects without chest pain (Group 1); gray solid line, non-diabetic subjects with chest pain (Group 2); black dotted line, diabetic subjects without chest pain (Group 3); black solid line, diabetic subjects with chest pain (Group 4).

**Table 3:** Hazard ratios (HR) of incident CAD events over 4 years of follow-up

	**Model 1**		**Model 2**		**Model 3**	
	**HR**	***P***	**HR**	***P***	**HR**	***P***
Non-diabetic subjects without chest pain (Group 1)	1		1		1	
Non-diabetic subjects with chest pain (Group 2)	2.768	<0.001	2.892	0.001	2.782	0.002
	(1.485 – 5.160)		(1.546 – 5.408)		(1.486 – 5.208)	
Diabetic subjects without chest pain (Group 3)	4.008	<0.001	3.253	0.001	2.626	0.005
	(2.079 – 7.727)		(1.671 – 6.334)		(1.333 – 5.172)	
Diabetic subjects with chest pain (Group 4)	13.220	<0.001	11.241	<0.001	8.539	<0.001
	(6.543 – 26.712)		(5.522 – 22.881)		(4.118 – 17.705)	

*Abbreviations*: CAD, coronary artery disease.

Model 1: No adjusting.

Model 2: Adjusted for age and sex.

Model 3: Adjusted for age, sex, bmi, hypertension, dyslipidemia, smoking history and family history of CAD.

## Discussion

In our study, among 8,574 subjects without a history of CAD, 0.8% and 2.2% of non-diabetic and diabetic subjects, respectively, reported experiencing newly developed CAD events during a 4-year follow-up period; these rates are concordant with those of the DIAD study [4]. Our results corroborate those of earlier reports indicating that subjects with diabetes mellitus have an increased incidence of cardiovascular events [1,14] and show that the presence of chest pain at baseline is significantly associated with an increase in future CAD risk of more than 2-fold in both non-diabetic and diabetic subjects.

Interestingly, diabetic subjects without chest pain had a similar CAD event rate to non-diabetic subjects with chest pain, implying that the results of clinical trials conducted in asymptomatic non-diabetic subjects are not applicable to asymptomatic diabetic subjects. The well-known clinical trials which showed that revascularization was not superior to medical treatment for stable CAD [6,15] included subjects with diabetes only 20–35% of the study population and those results should be carefully interpreted when applying them to diabetic subjects.

Although the Bypass Angioplasty Revascularization Investigation 2 Diabetes (BARI 2D) trial did not find any difference in cardiac outcomes between revascularization and medical treatment in the patients with diabetes, subgroup analysis showed that the prognosis of severe CAD lesions was better with revascularization treatment [5]. The survival of diabetic patients with silent ischemia is known to be related to the severity of CAD [16]. Considering the fact that small proportion of subjects with moderate or large perfusion defects underwent coronary angiography within 120 days after screening in the DIAD study [4], the benefit of screening might be underestimated in that study.

The present study also revealed that no baseline characteristics, except age in diabetic subjects, were significantly different between subjects with and without CAD, which corroborates the results of previous studies [2,3]. In contrast, the traditional risk factors for CAD such as age, obesity, and hypertension were significantly associated with future CAD event rates in non-diabetic subjects. Previous studies report that CAD risk indicators other than traditional risk factors for asymptomatic diabetic patients include autonomic neuropathy [2,17], retinopathy [18,19], and renal complications [20,21]. However, in the present study, we only had information on kidney function, and there was no difference in serum creatinine level or albumin excretion ratio with respect to CAD events in diabetic patients.

Improvements in the management of diabetic patients with multiple risk factors might be a reason for the lack of associations between metabolic risk factors and the development of CAD events. In the present study, 23.2% of diabetic patients had uncontrolled hypertension at baseline, which is somewhat lower than the 33% reported in the general population in the Korean National Health and Nutrition Examination Survey in 2001 [22] and the 31% reported in the DIAD study population [2]. Intensive intervention with multiple drug combinations produces sustained beneficial effects with respect to vascular complications and mortality rates from any cause and cardiovascular causes, respectively [23]. A recent US report demonstrated that the mortality rates among both American men and women with diabetes decreased substantially between 1997 and 2006, reducing the absolute difference between adults with and without diabetes [24].

However, further study to determine the high-risk population among asymptomatic diabetic patients is warranted by the fact that diabetic patients with silent ischemia have poor outcomes [25] and that the prognosis of severe CAD lesions is better with revascularization treatment [5]. Asymptomatic diabetic patients with a higher coronary disease burden suffer more future cardiac events than asymptomatic patients do [26,27].

The main limitation of our study is that CAD events were determined from questionnaires without objective confirmatory data. The presence or absence of chest pain was also determined from questionnaires, which might result in underestimation. The relatively short follow-up duration of the present study is also a limitation for investigating the CAD event rate. However, the prospective 4-year follow-up of a large community-based cohort means our results are stronger than those of other studies are. Furthermore, few studies have compared the impacts of chest pain on future CAD in those with and without diabetes.

## Conclusions

The CAD event rate of asymptomatic subjects with diabetes was comparable to that of non-diabetic subjects reporting chest pain. Considering the high risk of CAD in asymptomatic diabetic patients and morbidity and mortality due to CAD, more clinical trials aimed at formulating strategies to screen asymptomatic diabetic subjects should be carried out.

## Competing interests

We have no potential conflicts of interest to report.

## Authors’ contributions

BK wrote the manuscript and collected data. YK made substantial contributions to conception and design and KP contributed to the discussion and reviewed the manuscript. MM contributed to the discussion, and reviewed and edited the manuscript. All authors read and approved the final manuscript.

## Pre-publication history

The pre-publication history for this paper can be accessed here:

http://www.biomedcentral.com/1471-2261/13/87/prepub
